This article has been retracted.

# An Investigation of Electrospun *Clerodendrum phlomidis* Leaves Extract Infused Polycaprolactone Nanofiber for In Vitro Biological Application

**DOI:** 10.1155/2022/2335443

**Published:** 2022-07-09

**Authors:** Siranjeevi Ravichandran, Rajesh Jegathaprathaban, Jeyalakshmi Radhakrishnan, R. Usha, V. Vijayan, Aklilu Teklemariam

**Affiliations:** ^1^Department of Chemistry, Saveetha School of Engineering, Saveetha Institute of Medical and Technical Sciences, Saveetha University, Chennai 602105, Tamil Nadu, India; ^2^Department of Chemistry, SRM Institute of Science and Technology (SRMIST), Kattankulathur 603203, Kancheepuram (DT), Tamil Nadu, India; ^3^Department of Physics, Saveetha School of Engineering, Saveetha Institute of Medical and Technical Sciences, Saveetha University, Chennai 602105, Tamil Nadu, India; ^4^Department of Mechanical Engineering, K. Ramakrishnan College of Technology, Samayapuram, Trichy 621112, Tamil Nadu, India; ^5^Department of Mechanical Engineering, Faculty of Manufacturing, Institute of Technology, Hawassa University, Hawassa, Ethiopia

## Abstract

The in vitro antibacterial, anticancer, and antioxidant activities of a few plant extracts were widely known for decades, and they were used for application in the conventional way. Specifically, electrospun nanofibrous mats have recently exhibited great antibacterial, anticancer, and antioxidant activities. The herbal extracts infused into these formations are expected to have a more efficient and integrated effect on in vitro biological applications. The purpose of this study is to develop polycaprolactone- (PCL-) based nanofiber mats that are infused with a traditional plant extract using *Clerodendrum phlomidis* leaves to improve the synthesized nanofibers' antibacterial, anticancer, and antioxidant efficacy. This study examined the morphology, thermal properties, mechanical properties, structure, and in vitro drug release studies of electrospun nanofibers. Antibacterial, anticancer, and antioxidant activities of the electrospun nanofibrous mats were also studied. The HRTEM and FESEM pictures of PCL and PCL-CPM nanofibers provide that smooth, defect-free, and homogeneous nanofibers were found to be 602.08 ± 75 nm and 414.15 ± 82 nm for PCL and PCL-CPM nanofibers, respectively. The presence of *Clerodendrum phlomidis* extract in the electrospun nanofibers was approved by UV-visible and FTIR spectroscopy. The incorporation of *Clerodendrum phlomidis* extract to nanofiber mats resulted in substantial antibacterial activity against bacterial cells. PCL-CPM mats exposed to oral cancer (HSC-3) and renal cell carcinoma (ACHN) cell lines displayed promising anticancer activity with less than 50% survival rate after 24 h of incubation. 2,2-Diphenyl-1-picrylhydrazyl (DPPH) assay performed on PCL-CPM nanofibers revealed the antioxidant scavenging activity with maximum inhibition of 34% suggesting the role of the secondary metabolites release from scaffold. As a result, the findings of this study revealed that *Clerodendrum phlomidis* extract encapsulating PCL electrospun nanofibers has a high potential for usage as a biobased antibacterial, anticancer, and antioxidant agent.

## 1. Introduction

Natural plant extracts have recently gained a lot of popularity in medicine for the treatment and prevention of refractory and socially significant diseases [1–5]. This plant is represented by *Clerodendrum phlomidis* extract, which has a range of beneficial biological activities such as analgesic [6], antiamnestic [7], antiasthmatic [8], antidiarrheal [9], anti-inflammatory [10], antimicrobial [11], antifungal [12], antiplasmodial [13], antiviral [14], hypoglycemic [15], immunomodulator [16], and psychopharmacological [17]. *Clerodendrum phlomidis* extract has a low bioavailability due to its poor solubility in organic solvents, water low absorption, chemical instability, high metabolism, bodily fluids, and elimination from the human body. These defects can be overcome by combining *Clerodendrum phlomidis* extract in appropriate polymer nanofibers. Electrospinning is a cutting-edge development for producing micro- and nanofibrous mats from synthetic and natural polymers, which can include a wide range of natural medicines [18, 19].

Electrospinning is an efficient and relatively simple technique. This method involves a large surface area of nanofibers [20]. Many plant extracts, such as pineapple, *Centella asiatica, Garcinia mangostana, Rubus strigosus,* grape seed, and *Aloe vera*; essential oils; and gallic acids are incorporated into these electrospun nanofiber mats for biological uses [21–23]. Curcumin nanofibers are used in combination with PCL-cum Tracacon to treat bacterial and diabetic wounds. They noted the high mechanical strength of polycaprolactone and the good biological activity of these nanofibers, and their nanofiber mats are recommended for wound healing [24].

Many naturally occurring agents are effective in chemoprevention and chemotherapy in a variety of biochemical systems and animal models [25]. Recently, incorporation of natural plant extracts in nanofibers was studied for various biomedical applications. For example, chitosan-based electrospun nanofibers incorporated with a *Lawsonia inermis* (Henna) leaf extract have been administered to patients to improve antibacterial action and wound healing efficacy [26]. Similarly, the potential of curcumin-incorporated PCL/gum tragacanth electrospun nanofiber mats that heal diabetic wounds in rats has been noted and the use of these nanofibers in the treatment of such type of wounds is known to have enhanced the healing and recovery process [27]. Raghavendra et al. developed *Gymnema sylvestre*–loaded PCL/gelatin electrospun nanofibrous mats as a potential anti-infective wound dressing [28]. Suganya et al. prepared PCL/PVP nanofiber mats loaded with *Tecomella undulata* crude bark extract to investigate their antibacterial activity [29].

However, to the best of our knowledge, *Clerodendrum phlomidis* extract incorporated in polycaprolactone-based nanofibers designed for antibacterial and anticancer activity has not been reported yet. In this study, PCL-based electrospun nanofiber incorporated with *Clerodendrum phlomidis* methanol extract was synthesized for their potential application for antibacterial and anticancer activity. The morphology, thermal, and mechanical properties of the electrospun nanofibers mats were also investigated to support this objective.

## 2. Experimental Section

### 2.1. Materials

Sigma-Aldrich provided polycaprolactone (PCL), chloroform, and methanol (USA). All additional chemicals were purchased from licensed wholesalers. Fresh *Clerodendrum phlomidis* leaves were collected from the Thiruvarur district of Tamil Nadu, India. *Clerodendrum phlomidis* was identified and authenticated by Prof. P. Jayaraman of the Plant Anatomy Research Centre (PARC) in Chennai, Tamil Nadu, India.

### 2.2. Extraction of *C. phlomidis*

The powdered leaves (100 g) were successively extracted using *n*-hexane, ethyl acetate, and methanol by the Soxhlet apparatus for 8 hours. In a rotary evaporator, the extracts were evaporated to near dryness, dried into a fine powder with a lyophilizer, and stored below 10°C for further analysis.

### 2.3. Fabrication of CPM-Loaded PCL Nanofibrous Mats

The electrospinning of the PCL and PCL-CPM was performed using ESPIN-NANO V1 (Figure 1). PCL pellets were added to a mixture of methanol and chloroform (1 : 3 v/v) at room temperature and dissolved completely. To this solution, 6 wt% of sonicated CPM in methanol was mixed and the solution was stirred overnight. A 5 mL syringe with a 21 G needle was used to inject the solution. The electrospinning parameters such as the high voltage of 12 kV, the flow rate of 1 ml/h, and tip to target distance of 12 cm were employed. The nanofibers were deposited onto the aluminum-foil-wrapped grounded collector. To remove any remaining solvents from the nanofibers, they were processed in a vacuum dryer [30–32].

### 2.4. Characterization of PCL and PCL-CPM Nanofibers

The surface features and fiber diameter of PCL and PCL-CPM nanofibers were revealed using FEI Quanta FEG200 (FESEM). The determination of nanofiber diameter and standard deviation were done using ImageJ software. A high-resolution transmission electron microscope (JEOL Japan, JEM-2100 plus) at an implementing voltage of 200 kV was used for the experiment. Fourier transforms infrared (FTIR) analysis was assessed in the ALPHA-T-FT-IR Spectrometer. Thermal degradation analysis was done by performing differential scanning calorimetry (DSC) (TA Instruments, Waters, Austria, Q200). Thermal stability was examined in TGA : Q50 TA Instruments, Water Pvt. Ltd., India. The mechanical properties of nanofibrous mats were measured using Instron tensile tester (USA). The hydrophilic or hydrophobic nature of electrospun nanofiber mats was determined using VCA optimum surface analysis system (AST Products Billerica, MA).

### 2.5. In Vitro Drug-Releasing Profile

The nanofibrous mats were cut into 3 × 3 cm^2^ pieces. About 20 mg weight of the fiber mat was immersed in 10 ml of phosphate-buffered saline (pH = 7.4) containing vials. Vials were incubated at 37°C and at different time points; 200 *μ*L of the released solution was analyzed using UV-visible spectrophotometer. The experiments were carried out in triplicate, and the total percentage of CPM extract released from PCL-CPM nanofibers was calculated [3, 17].

### 2.6. Antibacterial Activity

The antibacterial activity of CPM-loaded PCL nanofibers was evaluated using disk diffusion assay against some commensal Gram-positive and Gram-negative bacteria. Briefly, bacteria suspension cultured in Mueller Hinton Broth (MHB) for 24 h was assessed to 0.5 McFarland standard. A 100 *µ*l of this adjusted culture was placed over sterile Mueller Hinton Agar (MHA) plates. Then nanofibers were cut into circular disks placed onto the agar plates and incubated for 24 hours at 37°C. The inhibitory zone formed was measured in millimetres. The studies were performed in duplicate [33, 34].

### 2.7. In Vitro Cytotoxicity Study

The cytotoxicity of the CPM extract, PCL, and PCL-CPM nanofibers was determined against oral cancer (HSC-3) and renal cell carcinoma (ACHN) cell lines. The samples were divided into three groups: (i) test cells (control), (ii) naive PCL nanofiber, and (iii) PCL-CPM nanofiber. Various nanofiber samples were added to 96 well plates containing 10 ml of phosphate-buffered saline (pH 7.4). Briefly, the HSC-3 and ACHN cells were seeded over the nanofibers and incubated overnight at 37°C to allow the cells to attach. To test cell viability, 1 mL MTT solution (5 mg·mL^−1^ in PBS) was added to the cultivated cells and was incubated for another 4 hours at 37°C. After removing the medium from each well, DMSO was added to solubilize the precipitate, and the absorbance was measured at 490 nm using a microplate reader (Microplate Reader 3550-UV, BIO-RAD). The relative cell viability rate was calculated by [OD]_test_/[OD]_control_ × 100 and the average value was obtained from triplicate [35–37].

### 2.8. Antioxidant Activity

#### 2.8.1. DPPH Radical Scavenging Method

The antioxidant activity of CPM and PCL-CPM nanofibers was analyzed using DPPH radical scavenging method. The DPPH scavenging behaviour was calculated using the approach examined by Aytac et al. with some changes. 1 mg of each PCL-CPM electrospun nanofiber sample was dissolved in 2 mL of freshly prepared DPPH ethanol solution (10^−4^ mol·L^−1^, 80 percent, v/v) [38]. Absorbance was measured using a BioMate-3 UV/Vis spectrophotometer (Thermospectronic, Handheld, AL, USA) at 517 nm. 0.1 mL of CPM solution (80%, v/v) was added with 2 mL of the newly prepared DPPH solution at various concentrations. The scavenging activity was determined using (1), where A_control_ and A_sample_ represent the absorption values of DPPH solution both with and without the presence of the sample, respectively.

(1) $$\begin{array}{c} \text{Antioxidant Activity}\left(\%\right)=\frac{A_{\text{Control}}-A_{\text{Sample}}}{A_{\text{Control}}}\times 100. \end{array}$$

## 3. Results and Discussion

### 3.1. Morphology and Spectroscopic and Thermal Properties of Nanofiber

The surface morphology of PCL and PCL-CPM nanofibrous mats was studied using FESEM (Figure 2) and HRTEM (Figure 3). The formed nanofibers were smooth, randomly oriented, and bead free. However, as seen in Figure 2(b), after PCL nanofibers were loaded with *Clerodendrum phlomidis* methanol extract, the surface morphology of PCL was not affected. The results indicated that the diameter of PCL nanofibers decreased from 617.91 ± 16 to 426.77 ± 14 nm after the addition of CPM extract (PCL-CPM nanofibers). It has been reported that as the conductivity and viscosity of the dope solution increase, the diameter of electrospun PCL nanofibers decreases. The presence of phytochemicals in the CPM extract, such as lupeol, alkaloid, phenol, flavonoid, and Clerodendrin-A, leads to reduced viscosity and improved conductivity of the resulting solution, in turn resulting in reduced diameter of the composite fiber. Similar observations have been made in studies in which the diameter of the fiber was highly impacted by its solution parameters. Hadisi et al. prepared PLA nanofibrous mats incorporated with various amounts (in percentage) of *Garcinia mangostana* extract. They found a moderate decrease in the fiber diameter when the concentration of *G. mangostana* increases due to a maximization in the conductivity of the electrospinning solution [39]. Hadisi et al. also assessed a decrease in the diameter of gelatin/oxidized starch hybrid nanofibers due to the reduction in the viscosity of the solution [40]. The TEM images of the prepared PCL and PCL-CPM electrospun nanofibers are revealed in Figure 3. It can be seen that the inner diameters of prepared PCL and PCL-CPM nanofibers were 602.08 ± 75 nm and 414.15 ± 82 nm, which are in agreement with the results obtained from SEM images. These observations clearly demonstrate the deposition of CPM extract–loaded PCL-CPM nanofibers within the wall surface presented in Figure 3(b).

The FTIR spectrum of the pure PCL and PCL-CPM electrospun nanofibrous mats is shown in Figure 4(a). Pure PCL showed the bands at 2947 and 2851 cm^−1^ are given to the symmetric and asymmetric stretching vibrations of CH_2_ groups. The peak at 1727 cm^−1^ is the C=O stretching vibration of the ester group, which appears with an intense, sharp peak and the CH_2_ bending vibration peaks occur at 1471 and 1386 cm^−1^. The absorption peaks centered at 1237 and 1051 cm^−1^ are clearly seen in the spectrum belonging to -C-O-C- asymmetric and symmetric stretching vibrations. The FTIR spectrum of the PCL-CPM nanofibers shows the C-H stretching vibration of alkanes occurring at 2947 cm^−1^ and the C=O stretching of the ketone group occurring at 1727 cm^−1^. The peaks at 830 and 1534 cm^−1^ are given to the primary amines (N-H bending) and nitro compounds (N-O asymmetric stretching). The presence of the stretching vibration of -C-O of primary and tertiary alcohol peaks at 1032 and 1168 cm^−1^ confirmed the successful incorporation of CPM extract into PCL nanofiber.

The UV-visible spectrum profile of PCL and PCL-CPM nanofibers is displayed in Figure 4(b). The profile showing the peaks at 229, 314, 406, 474, 508, 538, 602, and 666 nm was identified for PCL-CPM nanofibers, which correspond to the CPM confirming the loading of PCL-CPM nanofiber. The absorbance intensity of the PCL-CPM nanofiber increased, showing that the incorporation of CPM into the PCL nanofibers moves the absorption of PCL to a longer wavelength.

### 3.2. Thermal Analysis of PCL and PCL-CPM Nanofibers

Thermal degradation of PCL and PCL-CPM nanofibrous mats was studied by thermal gravimetric analysis (TGA).  Figure 5(a) shows the TGA image of PCL and PCL-CPM electrospun nanofibrous mats. As exhibited in the figure, for pure PCL electrospun nanofiber, the first stage of weight loss started at 330.42°C and the nanofiber entirely degraded at 474.0°C. However, two decomposition temperatures can be observed in Figure 5(a) at 270.92°C and 457.74°C, which are attributed to CPM extract and PCL. It can be seen that the exact mass losses of PCL and PCL-CPM nanofibers analyzed by TGA were approximately 96.63% (PCL) and 93.35% (PCL-CPM). These results show that *Clerodendrum phlomidis* methanol extract has been properly blended with PCL.

The DSC thermogram of electrospun nanofibers (Figure 5(b)) indicates sharp endothermic peaks at the temperatures of 65.91°C, 426.44°C, and 69.79°C, 428.97°C for PCL and PCL-CPM, respectively. This increased glass transition (*T*_*g*_) temperature of the latter which may be because of the addition of PCL polymer, improving the network structure between the polymers. The blending of PCL-CPM containing maximum amounts of OH group interacts with the phenolic OH and keto groups of *Clerodendrum phlomidis* extract. It can be seen that the higher endothermic peak suggests that the nanofibers have maximum stability at maximum temperature environments.

### 3.3. Contact Angle Studies

The water contact angles of PCL and PCL-CPM nanofibrous mats measured at 0 s and after 60 s of the water drop are shown in Figure 6 (Figure 6 reproduced from Ravichandran et al. [34]) and Table 1. As seen in Figure 6(a), the pure PCL nanofibrous mat had a contact angle of 137.44° at 60 s, which shows the hydrophobic nature of PCL. But the contact angle of the *Clerodendrum phlomidis* methanol extract incorporated PCL (PCL-CPM) was observed to be 94.22° at 0 s, which decreased to 45.81° after 60 s due to the presence of hydrophilic groups (Figure 6(b)). This enhanced hydrophilicity of PCL-CPM leads to better cell adhesion, better swelling, proliferation, and controlled drug release than PCL alone. The water contact angle results indicate that phytocomponents enhanced the wettability of nanofiber.

### 3.4. Mechanical Characterization

The mechanical strength of the PCL and PCL-CPM nanofibers was displayed in Figure 7(a) (Figure 7(a) reproduced from Ravichandran et al. [34]) and corresponding tensile strength, Young's modulus, and elongation at break are listed in Table 2. The mechanical properties of pure PCL nanofibers exhibited minimum tensile stain responding to plastic deformation of the nanofibers. However, when *Clerodendrum phlomidis* methanol (CPM) extract is incorporated into PCL nanofibers, the nanofibers lose their plasticity. The results show a significant decrease in tensile strength compared to pure PCL nanofibers. In general, decreasing fiber diameter will increase the strength of the fibers and tensile modulus, while increasing the nanofiber diameter will increase the strain of failure [41, 42]. The fiber diameter of PCL-CPM is small (426.77 ± 14 nm), showing densely packed fibrillar structures and more complications compared to multiple junctions and deep PCL fibers (617.91 ± 165 nm). Lim et al. also discovered that small diameter fibers with densely packed lamellae and fibers structures have a high molecular orientation, which boosts tensile strength and hence improves mechanical strength [43]. Taken together, our findings imply that adding the extract to PCL improves its mechanical qualities significantly, highlighting the extract's excellent reinforcing potential.

### 3.5. Drug Release Studies

The drug release profile of CPM extract from the PCL-CPM electrospun nanofibers mats is shown in Figure 7(b). The release of CPM extract from the PCL nanofiber is rapid in the first 5 h after immersion in PBS followed by a sustained release after 12 h, which indicates the diffusion of small molecules from the inner side of fibers. This could be possible because of the greater penetration of water molecules into nanofibers with a larger surface area-to-volume ratio and increased porosity. The CPM extract gets deposited in the pores of nanofibers, with an initial rapid release to the nanofibers and final release percentage reaching 40% within 3 days. The extended time after 3 days does not change the rate of release. Though there was no crystallite or precipitation seen in the buffer, hydrolysis of the compounds from the CPM extract is the limiting factor for drug release. The secondary metabolites of herbal extract are released initially from the outer surface of the fibers when they are in contact with water. Thus, functional groups of CPM extract from PCL nanofibers changed the hydrophobicity of fibers as it was confirmed from lowering of contact angle (see Table 1), which indicates that intermolecular interactions facilitate the drug release rate.

### 3.6. Qualitative and Quantitative Analysis of CPM Extract

Phytochemical analysis of CPM showed the presence of coumarin, amino acid, diterpene, flavonoid, alkaloids, phenol, glycoside, quinones, protein, saponin, terpenoid, and steroids (Table 3). In addition, carbohydrates and tannins are also present in methanol extract.  Figure 7(c) represents the total bioactive constituents present in the sample. Spectral studies of secondary metabolites using GC-MS analysis clarified the relative abundance of more than 45 components while being compared to NIST library search.  Figure 7(d) and Table 4 show the active principles with their molecular weight (MW), retention time (RT), molecular formula, and peak area percent. The most important compounds were 1,2,3-propanetriol (5.95%); 2-methoxy-3-methyl-butyric acid, methyl ester (1.45%); palmitic acid (4.18%), ethyl, 9-hexadecenote (1.17%); hexadecenoic acid, ethyl ester (14.43%); phytol (31.58%), linolenic acid (1.09%); ethyl (9Z,12Z)-9,12-octadecadienoate (3.19%); and octadecanoate, ethyl ester (1.04%).

### 3.7. Antibacterial Activity

Antibacterial activity is a significant component of any substance used in biomedical applications. Several biodegradable and biocompatible polymers have been chosen as a carrier for drugs. The bacteria in the first critical class were Gram-negative, which include *Escherichia coli*, and *Pseudomonas aeruginosa, Salmonella typhi,* and *Staphylococcus aureus* belong to the high-class category. Therefore, present investigations are centered on the new classes of antimicrobial agents from medicinal plants that could significantly reduce the infections of antibiotic-resistant bacteria.

The bioactive components present in *Clerodendrum phlomidis* possess antimicrobial activity as reported by a few researchers and were considered as a good candidate against multidrug-resistant clinical isolates [44–46]. Hence the natural antimicrobial compounds from the nanofiber nuclear layer have been studied against both Gram-negative and Gram-positive bacterial strains after assessing their programmed drug-releasing behaviour. The mechanism of the antibacterial activity of nanofibers electrospun mats is relatively complex and not well studied. Smaller nanofibers have higher antibacterial activity, providing increases to the bacterial membrane. The released plant extract interacts with the bacterial cell wall, causing changes in cell wall shape as well as an increase in cell infiltration or damage, which leads to cell death. Nanofibers made from the PCL-CPM extract exhibit a strong affinity for phosphorus and sulfur-containing biomolecules found in intracellular components (DNA bases, protein) and extracellular (membrane protein). These biocomponents have an impact on respiration, ultimately influencing cell survival and cell division [47–50]. The antibacterial activity of PCL and PCL-CPM nanofibrous mats was tested against Gram-negative and Gram-positive bacteria (Figures 8 and 9). The activity of extract-free PCL nanofiber scaffold against these bacteria was used as control. No zone of inhibition was detected for the PCL nanofibers without CPM extract-loaded at any point of the preset time points as shown in Figures 8(a)–8(d), respectively, whereas PCL-CPM nanofibers clearing the zone of inhibition were observed. The bacteria were *E. coli* = 18 mm, *S. typhi* = 14 mm, S. *aureus* = 17 mm, and *P. aeruginosa* = 19 mm, respectively. The bacteria zone of inhibition on the CPM extract was smaller than that on the PCL-CPM nanofibers at the studied time points. The results for the antibacterial activity of CPM extract incorporated in the nanofibers (PCL-CPM) showed an increase in such activity. These results indicate that PCL-CPM nanofiber mats have promising potential as effective wound dressing agents. The possible mechanisms of antibacterial activity of PCL-CPM nanofibers are diagrammatically represented in Figure 10.

### 3.8. Anticancer Activity

The cytotoxicity effects of PCL and PCL-CPM electrospun nanofibers mats were tested on two cancer cell lines of different lineages: HSC-3 (oral cancer) and ACHN (renal cell carcinoma) obtained from the Japanese Collection of Research Bioresources (JCRB) Cell Bank and the National Centre for Cell Science (NCCS), Pune, respectively. The cells were cultured in (DMEM) (Dulbecco's Modified Eagle Medium) containing 10% fetal bovine serum (FBS). Both cells were kept at 37°C for 24 h. In the case of control and without loaded *Clerodendrum phlomidis* extract PCL nanofibers, the drug-free samples did not show any cytotoxicity to the HSC-3 and ACHN cells up to 24 h (Figure 11 and 12). The cytotoxicity of PCL-CPM electrospun nanofibers against HSC-3 and ACHN cells displayed reducing cell viability with culture time. In the case of PCL-CPM nanofiber mats, all the samples showed decreasing cell viability with culture time. The PCL-CPM nanofibers mats inhibited cell growth at rates of 55% and 56% after 48 h of administration and an increasing tendency of growth inhibition was observed at 72 h. As can be seen, the cytotoxicity of CPM arises from its release from the PCL nanofibers. Furthermore, when compared to PCL nanofibers, PCL-CPM nanofibers revealed significantly higher cytotoxicity against HSC-3 and ACHN cell lines. The CPM incorporated PCL nanofibers exhibiting anticancer activity and thus representing the development of a novel CPM extract that can be used for localized treatment of cancer.

The mechanism that involves nanofibers' anticancer activity is generally complex. Nanofibers are phytocompound carriers that may also act as anticancer agents. Nanofibers have positive charges with opposite charges that are responsible for nanofiber uptake and internalisation, whereas cell membranes (cancer/normal) carry negatively charged components like lipids. The surface area of nanofibers has the greatest impact on cell internalisation. ROS production via the caspase cascade of apoptosis, DNA damage, and mitochondrial malfunction all contribute to cytotoxic action [36, 51].  Figure 13 depicts the various mechanisms of anticancer activity of PCL-CPM nanofibers in diagrammatic form.

Similarly, other studies have explored observations that studied the release of compounds with the incorporation of nanofibers. Young-Jin Kim et al. synthesized polyphenol-incorporated PCL nanofibers and found a slightly higher cytotoxic effect against MKN28 compared with PCL-polyphenol nanofibers. The released plant polyphenol is the main cause of EGCG and CA cytotoxicity [52].

### 3.9. Antioxidant Activity

The antioxidant activities of *Clerodendrum phlomidis* extracts have been associated with a variety of compounds that exhibit various reduction and radical quenching abilities, including 2,3-dihydroxypropanal, 2-methoxy-4-vinylphenol, 3,6,7-trihydroxy-2-(3-methoxyphenyl)-4*H*-chromen-4-one, caryophyllene, oleic acid, and eicosyl ester [53]. Flavonoids, phenolic acids, and their derivatives' antioxidant activity is impacted by their chemical structure, which is influenced not only by the location and number of hydroxyl groups, but also by the presence of certain compounds, such as conjugated double bonds in the C-ring with carbonyl groups or catechol in aromatic rings. Furthermore, the ability of polyphenolic compounds to act as antioxidants has been demonstrated to be dependent on the redox characteristics of their phenolic hydroxyl groups, as well as their propensity for electron delocalization through the chemical structure [54]. In addition, natural plant extracts exhibit antioxidant activities due to bioactive secondary metabolites by different mechanisms of action and potential synergistic interactions. It is also important to note the type of methods to assess the antioxidant ability. Among them, commonly used DPPH techniques have been widely employed for natural products [36]. Moreover, these methods have been used widely to study for electrospinning fibers [55, 56], active packaging films [57, 58], and nanoparticles [59]. Therefore, radical scavenging activity of the extract loaded on the scaffold was evaluated and related to the phytochemical activity.

Figure 14(a) shows the antioxidant activity of the solutions of CPM extract prepared by tested AO assays at various concentrations (mg_CPM_ kg^−1^) as a function of time. An increase in antioxidant activity was observed with increasing CPM extract concentration until a steady state was reached for approximately 300 min. These results demonstrated a direct correlation antioxidant activity of CPM extract solutions with active polyphenolic components such as flavonoids, tannin, and alkaloids components. Further to that, the other secondary metabolites identified in the CPM from GC-MS analysis are tetradecanoic acid, n-hexadecanoic acid, and hexadecanoic acid. These are known antioxidant compounds having redox properties because of their free radical absorption and neutralization reaction. Therefore, the presence of these compounds in the extract and thereafter in the scaffold is responsible for the multiple therapeutic properties as discussed in the earlier sections.

The antioxidant activity of PCL-CPM nanofibers with time for antioxidant activity is shown in Figure 14(b). As shown in Figure 14(a), increasing the amount of CPM in the PCL-CPM electrospun nanofibers resulted in an increasing pattern of antioxidant activity, as evidenced by the colour changes that occur based on CPM content in the nanofibers. The PCL-CPM electrospun nanofibers have shown AO, demonstrating the effective incorporation of CPM extract by electrospinning. Furthermore, with increasing CPM extract loading, the overall antioxidant activity of nanofibers expressed as *μ*mol_Trolox_ mg_fibre_^−1^ increased significantly (*p*0.05), which was directly related to the CPM extract content contained in the nanofibers. These results agree with the findings of other researchers who have detected similar associations between fiber antioxidant activity and the content of the active compound present in the materials. Aydogdu et al., for example, found that increasing gallic acid content in polymer formulations increased antioxidant activity of hydroxypropyl methyl cellulose/PEO fibers (Aydogdu et al). Similarly, when higher levels of rosmarinic acid were encapsulated, Vatankhah et al. seen higher antioxidant activity of cellulose acetate fibers. In addition, the AO of polymer fibers or sheets containing natural ingredients indicated for food packaging applications has been established by several scholars, and similar antioxidant behaviour was discovered when diverse natural extracts were used [60, 61]. The AO of 0.120 *μ*mol_Trolox_·mg^−1^ in PVA nanofibers containing rosemary extract [62], 0.013 *μ*mol_Trolox_·mg^−1^ in starch sheets infused ethanol extract (propolis), 0.005 *μ*mol_Trolox_·mg^−1^ in zein nanocomposite sheets containing pinhao extract, and 0.011 *μ*mol_Trolox_·mg^−1^ in chitosan sheets incorporated with extract (maqui berry) was revealed [63, 64].

## 4. Conclusions

In conclusion, we have described the most efficient and repeatable method of producing a drug delivery system based on polycaprolactone nanofibers containing bioactive compounds from *C. phlomidis* leaves. The surface morphology of nanofibers analyzed by FESEM and HRTEM showed that the proportion of *Clerodendrum phlomidis* extract affected fiber diameters, and the components in the extract reduced the diameter of the nanofiber, increasing the wettability. Antimicrobial and anticancer research studies are encouraging because of enhanced bioavailability through adsorption and diffusion of nanosize fibers. Antioxidative components present in the extract effectively inhibit the viability of cells in vitro in HSC-3 (oral cancer) and ACHN (renal cell carcinoma). Our results illustrate a promising use of PCL-CPM electrospun nanofibers as a nanoplatform for prolonged drug release for chemotherapy in the clinical treatment of cancer. CPM extract kept its similar bioactivity after being added to the polymer mixtures, despite the high voltage used during the electrospinning process. The design of formulations at room temperature may help to prevent and/or restrict the processes of thermal degradation of thermolabile compounds present in the CPM extract.

## Figures and Tables

**Figure 1:** Schematic diagram display electrospinning setup used to prepare CPM extract-infused PCL nanofibers (PCL-CPM nanofibers).

**Figure 2:** SEM images of electrospun nanofibers: (a)PCL and (b) PCL-CPM nanofibers. The fiber distribution is represented in the extreme right column.

**Figure 3:** TEM image of PCL and PCL-CPM nanofibers.

**Figure 4:** (a) FTIR and (b) UV-visible spectrum.

**Figure 5:** (a) TGA thermograms and (b) DSC thermograms.

**Figure 6:** Water contact angle for PCL (a_0s_–b_after60s_) and PCL-CPM (c_0s_—d_after60s_) (Figure 6 is reproduced from Kim et al. [36]).

**Figure 7:** (a) Mechanical properties. (b) Cumulative release profile. (c) Quantitative analysis of CPM extract and D. GC-MS analysis of CPM extract (Figure 7 is reproduced from Kim et al. [36]).

**Figure 8:** Antibacterial activity of extract (CPM), PCL and PCL-CPM nanofibrous mats: (a) *E. coli*, (b) *S. aureus*, (c) *S. typhi,* and (d) *P. aeruginosa*.

**Figure 9:** (a) *E. coli*, (b) *S. aureus*, (c) *S. typhi*, and (d) *P. aeruginosa*. Zone of inhibition with crude extract (*C. phlomidis*), PCL, and PCL-CPM nanofibrous mats.

**Figure 10:** A diagrammatic representation of the mechanisms of antibacterial activity of the nanofibers.

**Figure 11:** Cytotoxicity of the blank PCL and PCL-CPM nanofibers to the ACHN (renal cell carcinoma) cells. (a) Blank control, (b) 0% (blank PCL), and (c) PCL-CPM nanofiber.

**Figure 12:** Cytotoxicity of the blank PCL and PCL-CPM nanofibers to the HSC-3 (oral cancer) cells: (a) blank control, (b) 0% (blank PCL), and (c) PCL-CPM nanofiber.

**Figure 13:** A diagrammatic representation of the mechanisms of anticancer activity of nanofibers.

**Figure 14:** (a). Antioxidant activity of CPM extract at various concentration levels with time. (A) 100, (B), 200, (C) 300, (D) 400, and (E) 500). (b). Antioxidant activity of PCL-CPM electrospun nanofibers with time.

**Table 1:** Water contact angle of PCL and PCL-CPM nanofibers.

Sample	0 Second	60 Second
PCL	136.90 ± 0.46	135 ± 0.36
PCL-CPM	93.07 ± 0.52	45.81 ± 0.42

**Table 2:** Morphological characteristics and mechanical properties of PCL and PCL-CPM nanofibers.

Sample	Ave. fiber diameter (mm)	Tensile strength (MPa)	Elongation at break (%)	Young's modulus (MPa)
PCL	617.91 ± 165	2.2066 ± 0.543	131.153 ± 0.023	0.532 ± 0.519
PCL-CPM	426.77 ± 142	1.1626 ± 0.606	43.576 ± 0.625	27.24 ± 0.362

**Table 3:** Preliminary phytochemical screening of methanol extract of *Clerodendrum phlomidis*.

S. No	Phytochemicals	Methanol Extract
1	Alkaloids	+
2	Amino acids	−
3	Anthocyanin	−
4	Carbohydrates	+
5	Coumarin	−
6	Cardio Glycosides	−
7	Diterpene	+
8	Emodins	−
9	Flavonoids	+
10	Fatty acid	−
11	Leucoanthocyanin	−
12	Glycosides	+
13	Phlobatannin	−
14	Proteins	−
15	Phenols	+
16	Quinones	−
17	Saponin	+
18	Steroids	+
19	Tannins	+
20	Terpenoids	+

**Table 4:** GC-MS spectral analysis of methanol extract of *Clerodendrum Phlomidis*.

S. No	RT (min)	Name of the compound	Peak area (%)	Molecular weight	Molecular formula
1	3.05	Ethanedial dihydrazone	0.2	86	C_2_H_6_N_4_
2	3.15	1-Chloro-2-isocyanotoethane	0.33	105	C_3_H_4_ClNO_2_
3	3.70	2-Butene,1-methoxy-,(E)-	0.43	86	C_5_H_10_O
4	5.30	2,4-Pentadiensaecre,1-cyclopenten-3-on-1-yl ester	0.16	178	C_10_H_10_O_3_
5	5.53	1,2,3,-Propanetriol	5.95	92	C_3_H_8_O_2_
6	5.68	Phenol	0.56	94	C_6_H_6_O
7	5.78	Propane,1,1-dihydroxy-2-methyl-1,1-Diethoxy-2-methylpropane	0.38	146	C_8_H_18_O_2_
8	7.05	1,5-Heptadien-4-one,3,36-trimethyl-	0.14	152	C_10_H_16_O
9	7.30	Oxirane, phenyl-	0.35	120	C_8_H_8_O
10	7.77	2-Chloro-1-ethyl-1-methyl cyclopropane	0.14	118	C_6_H_11_Cl
11	7.95	Thymine	0.21	126	C_5_H_6_N_2_O_2_
12	8.97	Pentafluoropropionic acid, pentyl ester	0.16	234	C_8_H_11_F_5_O_2_
13	9.80	1,5-Anhydro-6-deoxyhexo-2,3-diulose	0.5	144	C_6_H_8_O_4_
14	10.73	Furan,2,3-dihydro-5-methyl-	0.13	84	C_5_H_8_O
15	10.80	1-Chloro-2-isocyanatoethane	0.23	105	C_3_H_4_ClNO
16	10.96	3,4-Anhydro-d-galactosan	0.19	144	C_6_H_8_O_4_
17	11.98	3-Pyridinecarboxylic acid	0.81	123	C_6_H_5_NO_2_
18	12.44	Benzeneacetic acid	0.26	136	C_8_H_8_O_2_
19	14.30	2-Methoxy-3-methyl-butyric acid, methyl ester	1.45	146	C_7_H_14_O_3_
20	14.65	Hexane,3-methoxy-3-methyl-	0.44	130	C_8_H_8_O
21	16.62	Cyclohexane, (2-methoxyethyl)-	0.37	142	C_9_H_18_O
22	16.76	Oxirane,2,2ؙ-(1,4-butanediyl)bis-	0.2	142	C_8_H_14_O_2_
23	17.34	Cyclohexanol,2,6-dimethyl-	0.21	128	C_8_H_16_O
24	19.25	2,6-Di-tert-butyl-4-methylphenol	0.82	220	C_15_H_24_O
25	19.96	1 (2H)-isoquinolinone	0.42	145	C_9_H_7_NO
26	21.98	Methyl beta-d-galactopyranoside	0.52	194	C_7_H_14_O_6_
27	21.98	L-(+)-Lactic acid, trimethylsilyl ester	0.14	162	C_6_H_14_O_3_Si
28	24.53	p-Toluic acid,2-octyl ester	0.24	248	C_16_H_24_O_2_
29	24.79	2-Propenoic acid,3 (3-hydroxyphenyl)- methyl ester	0.14	178	C_5_H_10_O_3_
30	25.05	Decanoic acid	0.31	172	C_10_H_20_O_2_
31	25.24	4,5-Heptadien-2-ol,3,3,6-Trimethyl-	0.15	154	C_10_H_18_O
32	25.65	Methyl benzoate	0.35	136	C_8_H_8_O_2_
33	26.45	p-Hydroxycinnamic acid, ethyl ester	0.29	192	C_11_H_12_O_3_
34	26.76	Z-4-Dodecenol	0.14	184	C_12_H_24_O
35	28.54	Hexadecanoic acid, methyl ester	0.31	270	C_17_H_34_O_2_
36	29.20	n-Hexadecanoic acid	4.18	256	C_18_H_32_O_2_
37	29.72	Ethyl,9-Hexadecenote	1.17	282	C_18_H_34_O_2_
38	29.87	Hexadecanoic acid, ethyl ester	14.43	284	C_18_H_36_O_2_
39	32.05	3,7,11,15-Tetramethyl-2-hexadecen-1-ol	31.58	296	C_20_H_40_O
40	32.39	9,12-Octadecadien-1-ol	0.53	266	C_18_H_34_O
41	32.49	9,12,15-Octadecatrienoic acid	1.09	278	C_18_H_30_O_2_
42	33.56	Ethyl (9Z,12Z)-9,12-octadecadienoate	3.19	308	C_20_H_36_O_2_
43	33.74	Octadecanoate, ethyl ester	1.04	312	C_20_H_40_O_2_
44	36.54	3-Hexenoic acid,5-hydroxy-2-methyl ester [R^*∗*^, R^*∗*^, (E)]	0.16	158	C_8_H_14_O_3_
45	37.83	Hexadecanoic acid,2-hydroxy-1-(hydroxy methyl) ethyl ester	0.14	330	C_19_H_38_O_4_

## Data Availability

The data used to support the findings of this study are included within the article and further data or information can be obtained from the corresponding author upon request.
